# Resveratrol Induces Apoptosis, Suppresses Migration, and Invasion of Cervical Cancer Cells by Inhibiting the Hedgehog Signaling Pathway

**DOI:** 10.1155/2022/8453011

**Published:** 2022-10-07

**Authors:** Jie Jiang, Zhenghua Liu, Xiuping Zhou, Fenglan Peng, Zhihui Wang, Feng Li, Ming Li

**Affiliations:** ^1^Department of Basic Medicine, Changsha Health Vocational College, Changsha, 410600 Hunan, China; ^2^Hunan Provincial Key Laboratory for Synthetic Biology of Traditional Chinese Medicine, Hunan University of Medicine, Huaihua, 418000 Hunan, China; ^3^Center of Trauma, The First Affiliated Hospital of Hunan University of MedicineHuaihua, 418000 Hunan, China; ^4^Department of Histology and Embryology, Hunan University of Medicine, Huaihua, 418000 Hunan, China

## Abstract

To investigate the effect and mechanism of resveratrol on the biological behavior of cervical cancer cells (HeLa cells), the apoptosis, migration, and invasion of HeLa cells were detected by flow cytometry, wound healing, and transwell assays. The expression levels of Hedgehog signal pathway proteins (smoothened (SMO), zinc finger transcription factors (Gli1), and sonic hedgehog homolog (Shh)) were detected by quantitative real-time PCR (qPCR) and western blotting. Compared with that control group, resveratrol (RES) significantly induced apoptosis, inhibited the migration and invasion of the HeLa cells. The expression of SMO, Gli1, and Shh were downregulated in the HeLa cells treated with RES. The Hedgehog agonist purmorphamine (PUR) reversed the RES-induced increase of apoptosis and reduction of migration and invasion in the HeLa cells. In conclusion, RES induced the apoptosis and suppressed the migration and invasion of HeLa cells by inhibiting Hedgehog signal pathway.

## 1. Introduction

Cervical cancer was a common malignant tumor in gynecology, and the incidence was second in gynecological malignant tumor [1] and increasing year by year [2]. With advances in the new diagnostic and therapeutic strategies, the mortality of cervical cancer had reduced. However, the treatment effect of patients with cervical cancer was still unsatisfactory. Therefore, it is urgent to search for new targets against cervical cancer, which are of great significance for improving the outcome of patients with cervical cancer.

Hedgehog signaling pathway was involved in the occurrence and development of tumors [3]. Some studies had investigated that Hedgehog signaling pathway was abnormally activated in cervical cancer [4]. Inhibition of Hedgehog signaling pathway could block the occurrence and progress of cervical cancer [5], which suggested that inhibiting Hedgehog was one of the strategies for treating cervical cancer.

Conventional treatments include surgery, chemotherapy, and radiotherapy for cervical cancer. The patients with early cervical cancer could be cured by surgery strategy [6], and those with advanced cervical cancer were treated with chemotherapy [7]. However, side effects on patients were inevitable due to the toxicity of the chemotherapeutic drugs. Therefore, the drugs with low toxicity and high efficiency had been explored for cervical cancer. In recent years, the traditional Chinese medicine had attracted attention for treatment of cervical cancer due to effective inhibition of proliferation and induction of apoptosis. Resveratrol (RES), a nonflavonoid polyphenol compound, was extracted from grapes, hellebore, and other plants [8]. Studies had shown that RES played a crucial role in anti-inflammatory [9], antioxidant, tumor prevention, and antiaging properties, but surprisingly, it had significant inhibitory effects on the progression of tumors [10]. A previous study had confirmed that RES alleviated breast cancer, ovarian cancer, and colon cancer by inhibiting the growth of tumor cells and promoting apoptosis [11]. It had been verified that RES blocked the proliferation and invasion of pancreatic and colorectal cancer cells by inhibiting Hedgehog signaling pathway [12]. RES had testified to have an anticervical cancer effect [13], but the specific mechanism is mystery. It remains unknown whether RES blocks the progression of cervical cancer through inhibiting migration and invasion, promoting apoptosis by weakening Hedgehog signaling pathway as same as pancreatic and colorectal cancer.

Here, we will explore the effect of RES on apoptosis, migration, and invasion of cervical cancer cells, and further clarify the potential mechanism of RES against cervical cancer. In this study, we verified that RES-induced apoptosis and suppressed migration and invasion by inhibiting Hedgehog signaling pathway in the HeLa cells, which provided a new theoretical basis for RES treatment of cervical cancer.

## 2. Materials and Methods

### 2.1. Cell Culture

Human cervical cancer cell (HeLa) was obtained from Nanjing University of Chinese Medicine and cultured in Dulbecco's Modified Eagle's Medium (DEME, Gibco, USA) with 10% fetal bovine serum (FBS, Gibco, USA) and antibiotics (100 mg/mL penicillin-streptomycin, Beyotime, China). HeLa cells were cultured at 37°C in a humidified incubator containing 5% CO_2_. The HeLa cells were treated with or without 40 *μ*mol/L RES (purity ≥ 99%, Aladdin Sigma, diluted in DMSO) [14] and Hedgehog pathway agonist purmorphamine (PUR, S3042, Selleck, USA).

### 2.2. Analysis of Cell Viability Using Cell Counting Kit-8 (CCK-8) Assay

HeLa cells were seeded into 96-well plate and were treated with different concentrations of Hedgehog signaling pathway agonist (PUR) for 48 h. Then, the cell viability was determined by CCK-8 assay (C0038, Beyotime, China) according to our previously published [15].

### 2.3. Assessment of Cell Apoptosis Using Flow Cytometry

HeLa cells were planted into 24-well plate. Cells were treated with or without RES and PUR at the confluence 50-60%. After 24 h, the cells were harvested and stained with Annexin V-FITC Apoptosis Detection Kit (AD10, Dojindo, Japan) in according the protocol of manufacture. Finally, the apoptosis of the cells was assessed using flow cytometry (BD, USA).

### 2.4. Determination of Cell Migration Using the Wound Healing Assay

HeLa cells were inoculated into 6-well plate. The cells treated with or without RES and PUR were cultured to 90% confluence, then, scratched uniformly with 10 *μ*L of tip. It was defined as 0 h when the cells were scratched. The area of scratches was photographed at 0 and 36 h or 48 h and analyzed by ImageJ software (Version 1.8.0, Softnic, USA).

### 2.5. Determination of Cell Invasion Using the Transwell Assay

The transwell chambers (BD, USA) were covered by Matrigel (BD, USA) for 3 h in incubator and arranged in the 24-well plate with medium containing 10% FBS. The HeLa cells were preincubated with or without RES and PUR, then, seeded into each chamber at concentration of 2 × 10^4^/200 *μ*L serum-free medium. The cells were incubated in the incubator for 24 hours and were fixed by 5% paraformaldehyde and stained with 0.1% crystal violet solution (Biosharp, China). The cells were scrubbed with cotton swab in the upper of chamber and randomly selected to photograph in the bottom of chamber. Finally, the number of cells was analyzed with ImageJ software.

### 2.6. Analysis of Hedgehog Signaling Pathway-Related Proteins (SMO, Gli1, and Shh) and Apoptotic-Related Proteins (Bax and Bcl-2) Expression by Quantitative Real-Time PCR (qPCR) and Western Blotting

The HeLa cells were treated with or without RES and PUR for 24 h; the cells were harvested to detect the expressions of SMO, Gli1, Shh, Bax, and Bcl-2, which were measured by qPCR and western blotting.

The total RNAs were isolated from HeLa cells using TRIzol reagent (Solarbio, China) in according to the protocol of manufacturer. The spectrophotometer (NanoDrop 2000, Thermo, USA) was used to measured concentration of total RNAs. The cDNA was obtained with All-One RT MasterMix Kit (abm, Canada) according to protocol of manufacturer. Finally, the expression *SMO*, *Gli1*, *Shh*, *Bax*, and *Bcl-2* were detected using qPCR MasterMix (MasterMix-S, abm, Canada) according to the protocol of manufacturer by CFX Connect™ Real-Time System (BIO-RAD, USA) with specific primers (forward primer: 5′-TGCTCATCGTGGGAGGCTACTT-3′, Reversed primer: 5′-ATCTTGCTGGCAGCCTTCTC-3′ for SMO; Forward primer: 5′-GACATACCCCACCTCCCTCT-3′, Reversed primer: 5′-ACTGCAGCTCCCCCAATTTT-3′ for Gli1; Forward primer: 5′-CAAGCAGTTTATCCCCAATGTG-3′, Reversed primer: 5′-TCACCCGCAGTTTCACTC-3′ for Shh; Forward primer: 5'-CATGTTTTCTGACGGCAACTT-3', Reversed primer: 5′-CCAGATCACGCCATTTCA-3′ for Bax; Forward primer: 5′-AAGAGCAGACGGATGGAAAAAGG-3′, Reversed primer: 5′-GGGCAAAGAAATGCAAGTGAATG-3′ for Bcl-2; Forward primer: 5′-AGAAACGGCTACCACATCCA-3′, Reversed primer: 5′-CACCAGACTTGCCCTCCA-3′ for 18S) under following parameters: predenaturation at 95°C for 10 mins; 40 cycles at 95°C for 15 s; 60°C for 1 min. The 18S was used as internal control. The expression of SMO and Gli1 was analyzed by 2^−ΔΔCt^ method [16].

The cells were lysed in RIPA buffer (P0013B, Beyotime, China) for 30 min on ice. The lysates were centrifuged at 4°C for 30 min at speed of 12,000 g. The supernatants were collected, and the proteins were determined using NanoDrop 2000 spectrophotometer. About 40 *μ*g proteins were separated by 10% SDS-polyacrylamide gel electrophoresis and transferred onto PVDF membranes (Millipore, USA). The membranes were incubated with 5% skim milk to block heterogenetic antigen at 4°C overnight, then, incubated with rabbit anti-Shh (1 : 1000, 20697-1-AP, Proteintech, China), rabbit anti-Bax (1 : 2000, 50599-2-Ig, Proteintech, China), rabbit anti-Bcl-2 (1 : 2000, 12789-1-AP, Proteintech, China), rabbit anti-SMO (1 : 500, ab235183, abcam, USA), rabbit anti-Gli1 (1 : 500, ab217326, abcam, USA), and rabbit anti-*β*-Actin antibodies (1 : 2000, AF5003, Beyotime, China) at room temperature (RT) for 2-3 h, following by incubating with HRP-labeled anti-rabbit IgG antibody (1 : 5000, A0208 Beyotime, China) at RT for 1-1.5 h. Finally, the proteins were visualized by chemiluminescence using gel imaging system (Chemidoc MP, Bio-Rad) and analyzed by ImageJ software.

### 2.7. Statistical Analysis

All data were from 3 independent experiments and presented as mean ± standard deviation. The SPSS23.0 and GraphPad Prism 8.0 software were used to analyze difference of the data. The difference between two groups was analyzed using independent *t-*test. The difference among groups was analyzed by Tukey's multiple comparisons of two-way ANOVA. The statistical difference was set as *p* < 0.05.

## 3. Results

### 3.1. RES Induced Apoptosis and Inhibited Migration and Invasion in HeLa Cells

To investigate the effects of RES on apoptosis, migration, and invasion, HeLa cells were treated with RES. Then, the apoptosis, migration, and invasion were, respectively, determined by flow cytometry, wound healing, and transwell assay. The apoptosis of the HeLa cells with DMSO (control group) was about 10%; however, the apoptosis of the HeLa cells with RES (RES group) was up to 20% (Figure 1(a)). As shown in Figure 1(b), the apoptosis of RES group was significantly higher than that of control group, which suggested that RES significantly promoted the apoptosis in the HeLa cells. After 48 h of the scratching, the scratch had healed completely in control group; however, the scratch was about 30-50% of the 0 h scratch in RES group (Figure 1(c)). The area of scratches in RES group was significantly wider than that in control group, which suggested that RES dramatically inhibited the migration of HeLa cells (Figure 1(d)). After 24 h of seeding, a large number of cells infiltrated the transwell chamber in control group, but a small number of cells infiltrated chamber in the RES group (Figure 1(e)). In other words, the count of cells in RES group was less than that in the control group, which revealed that RES notably suppressed the invasion of HeLa cells (Figure 1(f)).

### 3.2. RES Inhibited Hedgehog Signaling and Induced Expression of Apoptotic Proteins in HeLa Cells

To demonstrate the mechanism of RES regulation of cellular biological behavior, the expressions of Hedgehog signaling pathway related proteins (SMO, Gli1, and Shh) and apoptotic related proteins (Bax and Bcl-2) were detected by qPCR and western blotting. The expressions of SMO, Gli1, and Shh mRNAs were decreased in the RES group in comparison with that in the control group (Figure 2(a)). As shown in Figure 2(b), the expressions of SMO, Gli1, and Shh proteins were consistent with that of corresponding mRNAs. As shown in Figure 2(c), the expression of Bax mRNA was significantly increased in the RES group in comparison with that in the control group; the expression of Bcl-2 mRNA was obviously decreased in RES group relative to that in control group. The expressions of Bax and Bcl-2 proteins were consistent with those of Bax and Bcl-2 mRNAs (Figure 2(d)).

These results indicated that RES significantly inhibited Hedgehog signaling pathway, regulated apoptotic genes in HeLa cells.

### 3.3. PUR Reversed the Regulation of Apoptosis, Migration, and Invasion by RES in HeLa Cells

Previous experiments showed that RES could inhibit migration and invasion, induce apoptosis, and inactivate Hedgehog signaling pathway in the HeLa cells. To further clarify that RES regulates apoptosis, migration, and invasion through Hedgehog signaling pathway, HeLa cells were cotreated with or without RES and PUR. HeLa cells were treated with corresponding concentration of PUR. Then, the cell viability was analyzed by CCK-8 assay. As shown in Figure 3(a), the 50% effective concentration (EC_50_) was 1.079 *μ*mol/L based on viability of cells treated with PUR, and EC_50_ 95% confidence interval was 0.9401-1.237 *μ*mol/L. Therefore, cells were treated with 1 *μ*mol/L PUR for subsequent research.

Subsequently, the apoptosis, migration, and invasion of the cells were detected. The apoptosis of cells treated with RES was significantly increased in comparison with the control group, whereas, the apoptosis of RES + PUR group was decreased in comparison with that of RES group. The apoptosis was no observable difference between control group and PUR group; however, the apoptosis of RES + PUR group was higher than that of PUR group. The results of apoptosis had indicated that PUR partly inhibited RES-induced apoptosis (Figures 3(b) and 3(c)).

Since the scratches of the cells treated with PUR were 100% healed at 36 h, the images of scratch were photographed and analyzed at this time among groups. The area of scratch in the RES was obviously wider than that in the control group, while the area of scratch in the RES + PUR group was remarkably narrower than that in the RES group. The area of scratches in PUR group was 0, whereas, the area of scratch in the RES + PUR group was markedly wider in comparison with that in the PUR group. The results of wound healing had showed that PUR could reverse the inhibition of migration by RES in HeLa cells (Figures 3(d) and 3(e)).

As shown in Figures 3(f) and 3(g), the count of cells in the RES group was significantly less than that in the control group; nevertheless, the count of cell in the RES + PUR group was more than that in the RES group. The cell count of PUR group, which was same with that of the control group, was more than that of RES + PUR group. The results of transwell had suggested that PUR could reverse that suppression of invasion in HeLa cells.

There results showed that PUR could significantly reverse the regulation of apoptosis, migration, and invasion by RES in HeLa cells.

### 3.4. PUR Partly Abrogated the Downregulation of SMO, Gli1, and Shh Induced by RES in HeLa Cells

HeLa cells were coincubated with RES and PUR for 24 h. The expressions of SMO, Gli1, and Shh were analyzed by qPCR and western blotting. The Figure 4(a) showed that the expressions of SMO, Gli1, and Shh mRNAs in RES group were downregulated in comparison with that in control group; however, the SMO, Gli1, and Shh mRNA expression levels in the RES + PUR group were upregulated in comparison with that in the RES group. The mRNAs' expressions of SMO, Gli1, and Shh in the PUR group were increased in comparison with that in the control group, which indicated that PUR indeed activated the SMO, Gli1, and Shh mRNA expressions. The SMO, Gli1, and Shh mRNA expressions were downregulated in the RES + PUR group in comparison with that in the PUR group. Results demonstrated PUR partly abolished the downregulated of SMO, Gli1, and Shh mRNA expression levels induced by RES in HeLa cells. The expressions of SMO, Gli1, and Shh proteins were consistent with that of corresponding mRNAs, which displayed that PUR abrogated downregulated of SMO, Gli1, and Shh protein expression levels induced by RES (Figures 4(b) and 4(c)).

In summary, these results suggested that RES promoted apoptosis and inhibited migration and invasion in the HeLa cells; meanwhile, PUR could reverse regulation of biological behavior induced by RES in HeLa cells, which demonstrated RES-induced apoptosis and suppressed migration and invasion by inhibiting the Hedgehog signaling pathway in HeLa cells.

## 4. Discussion

Cervical cancer, which is one of the most frequent tumors in females, was the second leading cause of gynecological cancer-related mortality. Recurrence and metastasis were the main reasons for death in cervical cancer patients [17]. The treatment of cervical cancer mainly included surgery, chemotherapy, and radiotherapy. Although radical hysterectomy was feasible for early cervical cancer, radiotherapy or chemotherapy was feasible for local progression or advanced cervical cancer; however, about 50% of patients still experienced progression of cervical cancer due to drug resistance during treatment [18]. Although the research on the pathogenesis of cervical cancer had made some progress, there was still a lack of effective predictors and individualized alternative treatment. Therefore, it is necessary to further study the biological characteristics and medical intervention of cervical cancer in order to obtain better clinical treatment.

Invasion and metastasis of cancer cells were a complex process involving many factors, including the detachment of cancer cells from the primary site, degradation of the extracellular stroma through the secretion of matrix metalloproteinases, penetration of blood vessels and lymphatic walls, and finally the formation of new neoplasm in distant areas [19]. Although there were many researches on apoptosis, invasion, and metastasis of cervical cancer, the specific mechanism of progress of cervical cancer had not been completely clarified.

Hedgehog signaling pathway is a highly conserved signaling pathway that regulates embryonic development, cell growth, and differentiation after embryonic formation [20]. Hedgehog signal pathway mainly includes Shh, patched transmembrane protein receptor (Ptch), SMO, and zinc finger transcription factor protein (Glioma-associated oncogene transcription factors, Gli1, Gli2 ,and Gli3). The SMO, Gli1, and Shh played a crucial role in the Hedgehog signaling pathway on the progress of cancer. The SMO transduced signals to other proteins by interacting with Ptch, and abnormal expression of SMO promoted the cancer progression [21]. Gli1 was activated by Hedgehog signal transduction cascade, which regulated proliferation of cells [22]. Studies had showed that Gli1 was abnormally expressed in a variety of tumors [23] and suppression of Gli1 inhibited proliferation and migration of cancer cell [24]. Shh was abnormally elevated in various cancers and could serve as a potential biomarker to predict poor prognosis [25]. Downregulation of Shh could effectively inhibit progression of cancer [26–28]. It was verified that abnormal activation of Hedgehog pathway could lead to a variety of malignancies, including cervical cancer [29]. Kotulak-Chrzaszcz et al. had shown that SMO, Gli1, and Shh could promote progression of cervical cancer, but no drugs targeting SMO, Gli1, and Shh were approved for prevention and therapy of cervical cancer [30].

After the prevalence of COVID-19, traditional chinese medicine has become the focus on treatment of disease, including cancers. RES, a nonflavonoid polyphenol compound extracting from medicinal and edible homologous plants, had attracted attention on inhibition of tumor [31]. Studies had shown that RES had antioxidant and anti-inflammatory effects [32], and significantly inhibited the growth and migration of lung cancer, breast cancer, glioma, liver cancer, kidney cancer, and other tumors [31]. Our results had shown that RES induced apoptosis and antagonized the migration and invasion of HeLa cells, which was consistent with previous research confirming that RES could induce apoptosis and arrest migration and invasion through regulating different signaling pathways or genes, such as STAT3 signal pathway [33], FOXO3a [14], AHR [34], and RAD51 [35].

It was demonstrated that RES inhibited the malignant characteristics of pancreatic cancer cells [36] and renal cancer stem cells [37] by blocking Hedgehog signaling pathway. Our results had showed that RES significantly downregulated the expression levels of SMO, Gli1, and Shh in the Hedgehog signaling pathway of HeLa cells. To further prove that RES was closely related to Hedgehog on anticervical cancer. PUR, Hedgehog pathway agonist, was used to verify that RES promoted apoptosis and inhibited migration and invasion by blocking the Hedgehog pathway. The HeLa cells were treated with PUR, then, the apoptosis, migration, and invasion were detected. Surprisingly, the migration was promoted in the HeLa cells treated with PUR in comparison with that in the control group; however, the apoptosis and invasion in the PUR group were consistent with those in the control group. Interestingly, our studies had verified that PUR reversed the RES-induced increment of apoptosis and decreased of migration and invasion in the HeLa cells. It was wondering whether PUR effectively activated the Hedgehog signaling pathway. The results of qPCR and western blotting had showed that PUR could upregulate the Shh, SMO, and Gli1 expression, which suggested that PUR indeed activated the Hedgehog signaling pathway. Many studies had shown that activation of the Hedgehog signaling pathway could accelerate the progression of various tumors, and blocking this pathway was a new strategy for the treatment of tumors [38–41]. PUR-induced activation of Hedgehog signaling pathway could not promote the malignant characteristics of cervical cancer cells in our studies, which seemed to contradict previous researches. We speculated that the possible reason was as follow: Hedgehog signaling pathway had been abnormally activated in cervical cancer cell, which resulted in increment of malignant characteristics. Due to intrinsic Hedgehog signaling pathway activation, the malignant characteristics were not promoted after reactivating signaling pathway by PUR in the HeLa cells. Nevertheless, our results had also showed that PUR reversed the downregulation of SMO, Gli1, and Shh expression levels induced by RES, and partly abolished RES-induced increment of apoptosis and reduction of migration and invasion, which further confirmed that RES inhibited the progression of cervical cancer by inactivating the Hedgehog signaling pathway.

## 5. Conclusion

In conclusion, this study had shown that RES could induce apoptosis and suppress migration and invasion in the cervical cancer cell. RES could downregulate the expression of SMO, Gli1, and Shh. PUR partly abrogated inactivation of Hedgehog signaling, resulting in reverse the regulation of apoptosis, migration, and invasion induced by RES in HeLa cells; however the underlying molecular mechanism will be further investigated in vitro and in vivo. Regardless, these results provided a new therapeutic strategy for RES in the treatment of cervical cancer.

## Figures and Tables

**Figure 1:** RES promoted apoptosis and inhibited migration and invasion in HeLa cells. HeLa cells were treated with or without RES for 24 h (transwell assay) or 48 h (wound healing assay); the apoptosis (a and b), migration (c and d), and invasion (e and f) were, respectively, analyzed by flow cytometry, wound healing assay, and transwell assay. All date was from 3 independent experiments (^∗^*p* < 0.05, *t*-test). Control (Ctrl): HeLa cells were treated with DMSO; Resveratrol (RES): HeLa cells were treated with resveratrol (RES).

**Figure 2:** RES regulated the expression of Gli1, SMO, Shh, Bax, and Bcl-2 in HeLa cells. Cells were treated with or without RES for 24 h; the qPCR and western blotting were performed to analyzed the expression of Hedgehog signaling pathway-related genes (SMO, Gli1, and Shh (a and b)) and apoptotic-related genes (Bax and Bcl-2 (c and d)) in the HeLa cells. All date was from 3 independent experiments (^∗^*p* < 0.05, *t*-test). Ctrl: HeLa cells were treated with DMSO; RES: HeLa cells were treated with RES.

**Figure 3:** PUR reversed increase of apoptosis and decrease of migration and invasion in the HeLa cells. The cells were treated with or without RES and PUR for 24 h or 36 h. (a) The EC_50_ of PUR was calculated according to viability of cells by CCK-8. The apoptosis (b and c), migration (d and e), and invasion (f and g) of cells were, respectively, detected by flow cytometry, wound healing, and transwell assay. All date was from 3 independent experiments (^∗^*p* < 0.05, Tukey test). Control (Ctrl): HeLa cells were treated with DMSO; RES: HeLa cells were treated with RES; PUR: HeLa cells were treated with PUR; RES + PUR: HeLa cells were cotreated with RES and PUR.

**Figure 4:** PUR-inhibited downregulated the expression of SMO, Gli1, and Shh induced by RES in HeLa cells. Cells were treated with DMSO or RES or PUR or RES and PUR for 24 h; the expressions of Gli1, SMO, and Shh were analyzed by qPCR (a) and western blotting (b and c) in the HeLa cells. All date was from 3 independent experiments (^∗^*p* < 0.05, Tukey test). Control (Ctrl): HeLa cells were treated with DMSO; RES: HeLa cells were treated with RES; PUR: HeLa cells were treated with PUR; RES + PUR: HeLa cells were cotreated with RES and PUR.

## Data Availability

The data used to support the findings of this study are included within the article. Raw data are available from the corresponding author on reasonable request.
